RETRACTED

# The Influence of College Sports Services on Sports Behavioral Intentions: A Mediation Model Based on Satisfaction and Involvement

**DOI:** 10.1155/2022/2156128

**Published:** 2022-08-16

**Authors:** Zixiang Zhou, Ronghui Yu, Hao Cui, Yinggang Chen, Yixiang Li

**Affiliations:** ^1^Hoseo University, Asan-si 31066, Republic of Korea; ^2^College of Physical Education, Hunan University of Science and Technology, Xiangtan, Hunan 411201, China

## Abstract

To learn more about the impact of college sports services on student sports activity intentions, as well as the function of pleasure and involvement as a mediating factor in this process. According to the nature of the service, this study separates college sports services into basic and advanced sports two types, selects 482 students from five institutions in Hunan Province for a questionnaire survey based on spatial dimensions, and analyzes the data using a structural equation model. The findings show that (1) there is a positive correlation between college students' perception levels of basic and advanced sports services (*p* = 0.01); (2) perception of basic sports services is closely related to cognize involvement (*r* = 0.717), and perception of advanced sports services is closely related to affective involvement (*r* = 0.830); and (3) perception of basic sports services is closely related to cognize involvement (*r* = 0.717). (3) Satisfaction and involvement show a substantial mediation effect between sports service and sports behavioral intention, with involvement having a bigger influence on sports behavioral intention (effect percent = 52.63%) than satisfaction. (4) Advanced sports services are easier to improve students' behavioral intentions than basic sports services in a comparison of the two categories of college sports services. To summarize the findings of the four studies, it can be seen that ensuring the balanced development of basic and advanced sports services, adjusting service content to increase student involvement, and improving resource allocation to advanced sports service content are all effective ways to strengthen students' sports behavioral intention in the service strategy.

## 1. Introduction

The demand for sports services is increasing daily along with the interest that people have in participating in sports activities. In September 2019, the General Office of the State Council published “Opinions on Promoting National Fitness and Sports Consumption to Promote the High-Quality Development of the Sports Industry.” The sports services sector is expected to grow at a 60 percent yearly rate. Under government guidance, a number of sports service businesses have seen their growth accelerate recently, and the growth of college sports services has also been actively promoted. The overall quantity of sports resources available, however, limits the growth path of collegiate sports services, unlike public and commercial sports services with stated goals. Striking a balance between the two development strategies of enhancing sports service quality and building out sports service infrastructure is difficult. To meet the expanding demand for sports services, the issue of how to wisely allocate the limited sports service resources has emerged. According to many academics, the solution to this issue lies in developing targeted growth plans that are based on the particular sports service requirements of student groups. This study aimed to advance students' sports-related behavior as a practical goal in order to further investigate the impact of different kinds of college sports service content on students' sports-related behavior. Depending on the type of service, college athletic services are divided into basic and advanced sports services. Using a structural equation model, this study investigates the effects of two tiers of basic and advanced sports service on college students' desire to participate in sports.

RETRACTED

## 2. Concept Definition and Model Construction

### 2.1. Concept Definition

#### 2.1.1. Division of College Sports Services and Service Levels

The content of this survey on sports services in colleges and universities includes student physical health testing and sports facilities, sports organizations, sports activities, and sports equipment. Depending on the services offered, it is divided into two levels: basic sports services and advanced sports services. They are attached to one another. This is shown in Figure 1. The goal of the basic sports service is to maintain students' developing sports behaviors, whereas the goal of the advanced sports service is to raise the level of students' sports behaviors. In the plane dimension, basic sports service content incorporates advanced service material. The improvement and expansion of fundamental sports services in three dimensions are a component of advanced sports services. They all work together to form the framework for the spatial growth of college athletic services.

#### 2.1.2. Satisfaction of College Sports Service

Satisfaction is typically employed as a quantitative indicator to describe the comprehensive level of public sports services in research on public sports services. It refers to the public's subjective judgment of the quality of public sports services. Unlike other objective quality evaluation variables with survey limitations, satisfaction as a subjective evaluation variable can indirectly reflect the psychological expectations and actual needs of research subjects for service content and has better predictive validity for behavioral intentions [1]. Because the study's objective object is college sports services, which are split into basic and advanced sports services based on the nature of the services, the satisfaction response direction will no longer be limited to the field of service quality. According to satisfaction theory, whether the provision of service content satisfies individual expectations reflects satisfaction with basic services. If the supply quality of service content fulfills individual expectations, satisfaction with advanced services can be measured. The twofold standard of quantity and quality at the same time will indicate the total satisfaction of the service [2]. As a result, college sports service satisfaction will be defined as the subjective satisfaction of students with their college sports services in this study.

RETRACTED

#### 2.1.3. Involvement of College Sports Services

The term “involvement” refers to a psychological notion. This measure is commonly used in public service research to reflect the people's interest and passion for public services [3, 4]. The term “involvement” refers to a psychological notion. This measure is commonly used in public service research to reflect the people's interest and passion for public services. When employed as an intermediary variable in a service model, the degree of engagement can be used to measure the degree of demand for service content among the target population [5]. Furthermore, service involvement can be separated into two categories: cognitive involvement and affective involvement [6]. The reasonable cognitive state of the individual to the service, such as the rational cognition of the importance of the service content and the importance of the service content to sustain their own behavior for a long time, is one of them. Emotional engagement is linked to an individual's emotional state throughout the service, such as the emotional and spiritual feeling of the service content, as well as if the service content can elicit a positive emotion. To represent students' impressions of the content of these two different levels of sports services, the measurement of college sports service involvement in this study will focus on students' cognitive and affective involvement in basic and advanced college sports services. Cognition and emotional feelings are both important.

### 2.2. Model Construction

#### 2.2.1. The Impact of College Sports Services on Satisfaction and Involvement

From the perspectives of service quality and service content, the impact of service on satisfaction must be examined. First, according to [1], individuals' perceptions of service quality have a considerable impact on their satisfaction with service content, and perceived service quality has a favorable impact on satisfaction. Conclusions are applicable to several service kinds. Reference [7] splits the elements of community sports service into two types: core sports service provision and peripheral sports service provision in a research of sports service and satisfaction. This reveals that the core sports service provision content, which is dominated by sports facilities and institutions, has a favorable impact on sports service satisfaction, while the model route shows that volunteer-based peripheral sports service provision has no significant effect. Although the service must have a positive impact on satisfaction as a whole, the impact weight of different service components on satisfaction varies, which must be confirmed in the model based on the specific circumstances.

RETRACTED

From the perspectives of service demand and emotional motivation, the impact of service on involvement must be examined. The impact of service content on the degree of individual engagement was demonstrated in a study on the degree of audience involvement in advertising services by comparing the degree of audience involvement under different advertising contents. Reference [8] argues that when the content of the service is aligned with the individual's wants, it will boost the individual's cognitive engagement state at the level of service demand. The individual's attention to the service will be more focused at this time, and the rate of utilization and passion for the service content will also rise. The degree of match between the service content and the individual demands is thought to have a favorable effect on cognitive participation. At the level of emotional motivation, [9] argues that if the service's content causes the individual to experience pleasant emotions such as excitement and pleasure, it will increase their emotional engagement state. The individual's intention to use the service will be enhanced at this time, and their inclination to utilize the same service again in the future will also rise.

As a result, this study presents the following hypotheses based on the examination of the aforementioned connected ideas and the findings of similar investigations.

  H1: College sports services have a positive impact on involvement
  H2: College sports service has a positive impact on satisfaction

#### 2.2.2. The Effect of Satisfaction on Involvement

There is a clear link between satisfaction and participation. In service research, however, the degree of engagement, as a gauge of passion, can only explain an individual's attitude toward the service content, and it does not have a substantial impact on satisfaction on its own. Zhang Chonghui summarized past research in the field of consumer services on the degree of engagement and satisfaction, concluding that a high level of involvement does not always imply happiness with the service. Despite the notion that the one-way influence of engagement on satisfaction is restricted in diverse contexts, the effect of satisfaction on engagement has been established across multiple service categories, contradicting this conclusion. High audience satisfaction with commercials can boost engagement and motivate them to actively explore for information relating to advertised products, according to research on advertising services [10]. The conclusion of a related study on leisure sports services is that satisfaction has a positive impact on the degree of involvement and that those who are satisfied with sports services are more likely to be interested in and enthusiastic about leisure sports activities [11].

RETRACTED

As a result, this study presents the following hypotheses based on the examination of the abovementioned ideas and the findings of similar investigations.

  H3: Satisfaction has a positive effect on involvement

#### 2.2.3. The Influence of Involvement and Satisfaction on Sports Behavioral Intention

Individuals' service quality, expectations, cognition, and excitement are all reflected in their involvement and satisfaction. The favorable impact of the two on behavioral intentions can be shown in a variety of ways, including longer immersion intentions and more frequent participation intentions. This law also applies to the intentions of athletic behavior. Escart (2001) found that contentment has a favorable impact on sports behavioral intentions in his study of physical education services [12]. The influence of satisfaction on participants' intention to reexperience in the future was revealed in Shonk and Chelladurai's study on sports tourism [13]. In a study on skiing conducted by Kouthouris, the predictive effect of involvement on willingness to continue participation was proven [14].

As a result, this study presents the following hypotheses based on the examination of the aforementioned connected ideas and the findings of similar investigations.

  H4: Involvement has a positive effect on sports behavioral intention
  H5: Satisfaction has a positive effect on sports behavioral intention

#### 2.2.4. Hypothetical Model Construction (as Shown in Figure 2)

## 3. Research Objects and Methods

### 3.1. Research Objects

Hunan Province, one of China's 23 provinces, contains 13 prefecture-level cities and 106 colleges and universities, as well as a permanent population of 66.4449 million people and a 1.71% illiteracy rate. The entire population is large, and the educational level is high. This study employs the intentional sampling approach and the geographical dimension as the sample basis to select five prefecture-level cities (Changde City, Yongzhou City, Huaihua City, Zhuzhou City, and Xiangtan City) as the research region to assure the generalizability of the research conclusions. Simultaneously, the following is the decision reasoning for picking representative universities suitable for data gathering in the research area:

1. The selected university's quantity of sports service facilities matches the research requirements
2. The selected university's amount of sports services matches the research standards
3. Students at a few colleges have agreed to help with data collection

From the universities that satisfied the above three criteria, five representative universities were chosen for questionnaire distribution. The table below shows the total number of valid questionnaires recovered, as shown in Table 1.

RETRACTED

### 3.2. Research Methods

#### 3.2.1. Questionnaire Design

Table 2 lists the study's research variables and measurement parameters. The questionnaire design of the three elements of involvement, satisfaction, and behavioral intention, for example, is based on Park and Young, Rloliver, and Ajzen research, with only minor adjustments to the measurement content [6, 15, 16]. However, the sports service questionnaire has undergone significant revisions. The original reference scale (Zhou, 2019) has two subdimensions and five items for core and peripheral service provision, which are used to depict community sports from an individual's subjective standpoint. Service delivery status: the information has been altered to some extent because the survey's subject is college sports services. The specific adjustments include reorganizing the subdimensions, splitting the service content into two categories, basic and advanced, based on the nature of the differences, and increasing the number of measurement items from five to seven (sports facilities, sports organizations, sports activities, etc.). Complete coverage of key aspects of collegiate sports services, allowing it to represent the current state of the industry, is shown in Table 2.

#### 3.2.2. Questionnaire Reliability and Validity Test

The reliability and validity of this study were tested using SPSS statistical software, and the results are presented in the table below. The Cronbach coefficient was used to assess the reliability. The overall reliability may be judged to fulfill the demand criterion because all values were more than 0.7. Factor analysis was employed to test the validity of the study. The KMO values were all larger than 0.7, which matched the criteria for factor analysis, and each item's factor loading was greater than 0.5, with a total explained variance of more than 50%. Overall, the validity can be said to fulfill the demand standard, as shown in Table 3.

RETRACTED

## 4. Findings

### 4.1. Correlation Analysis

Table 4 shows the findings of the Pearson correlation analysis results. All of the variables in this study have a substantial positive correlation, and the collinearity statistics demonstrate that there is no serious multicollinearity between the data, indicating that the research hypothesis is originally established in the correlation verification. It is important to note that the correlation between the two variables of basic sports service (BSS)-advanced satisfaction (ASAT) and advanced sports service (ASS)-basic satisfaction (BSAT) is just 5%. As a result, the relationship between different categories of satisfaction and service content needs to be proved further, as shown in Table 4.

### 4.2. Model Fit Test

AMOS statistical software was utilized to test the model fit in this study.  Figure 3 depicts the model's path, while Table 5 lists the fitting indices derived from confirmatory analysis. The TLI, IFI, CFI, and NFI values are all greater than 0.9, whereas the SRMR and RMSEA values are all less than 0.08. It can be determined that the model's and data's fitting degree matches the requirements, and the fitting effect is satisfactory, as shown in Table 5.

### 4.3. Model Path Analysis

The model's path test results are provided in Table 6, and all routes reach the significant level of *P* = 0.001, indicating that the model accepts all of H1-H5's predicted paths. The influence of participation on sports behavioral intention (*β* = 0.644) is stronger than that of satisfaction (*β* = 0.362), as shown by a comparison of path coefficients in the model. There is no statistically significant difference between the influence of sports service on satisfaction (*β* = 0.509) and involvement (*β* = 0.553), as shown in Table 6.

### 4.4. Analysis of Mediation Effect

This study employed the PROCESS plug-in in SPSS statistical program to conduct Bootstrap analysis to further investigate the function of satisfaction and involvement as mediating factors in the model. We may estimate the influence of the two on sports behavioral intention by comparing the proportion of the total effect in the analysis results.  Table 7 shows the specific analysis results. It is clear that satisfaction and participation both play a role in mediating the relationship between sports services and sports behavioral intentions, with involvement slightly outperforming satisfaction in the effect ratio. The influence of involvement as a mediating variable appears to be slightly stronger than that of satisfaction, but the difference between the two only varies by 5%, and the difference is minor, as shown in Table 7.

RETRACTED

## 5. Discussion

### 5.1. Correlation between Advanced and Basic Sports Services

The correlation analysis finds a connection between sophisticated sports services and fundamental sports services (*P* = 0.01). The mechanism of this association can be seen as a representation of the internal consistency of the sports service as a whole from the perspective of subjective perception. The shortest wood plank among them all determines the barrel's capacity in the case of the barrel effect. College students' opinions of sports services are another issue that needs to be addressed. Sports services' overall reputation will suffer as a result of the relatively frail connections between advanced and basic sports services. This means that to invest in, develop, and offer sports programs in colleges and universities, a relative balance between the two levels must be struck and neither level may be overly favored. In particular, when sports services are being operated, there should be a coordinated interaction between advanced and basic sports services. If they are not balanced, students will have negative opinions of each one of them, which will harm the assessment of sports services as a whole.

### 5.2. The Effect of Advanced and Basic Sports Services on Satisfaction and Involvement

The model path analysis concludes that the route coefficients of overall satisfaction and involvement in sports services are extremely similar (*β* = 0.509; *β* = 0.553). This conclusion can be explained by the fact that both belong to subjective cognitive variables and reflect similar content when the content of all sports services is examined as a whole. However, as a result of the correlation study, it is clear that the degree of influence of different sports service levels on satisfaction and involvement varies greatly. Basic sports service and cognitive involvement are closer (*r* = 0.717), while advanced sports service and affective involvement are closer (*r* = 0.830). Advanced and basic sports service and associated satisfaction are also closer (*r* = 0.830). The correlations were tighter (*r* = 0.624; *r* = 0.680), and the non-corresponding satisfaction correlation was only significant at the 5% level (*P* = 0.01*, P* = 0.05). There is a distinct difference in the functions performed by the two in the influence path, as can be observed. Using modern sports services as an example, it can have a direct impact on emotional and cognitive involvement, as well as amplify the good effect on affective involvement.

RETRACTED

### 5.3. The Effect of Satisfaction and Involvement as Mediating Factors on Sports Behavioral Intention

The findings of a Bootstrap analysis of the influence paths of satisfaction and involvement demonstrate that both have a positive mediation effect on the path from sports service to sports behavioral intention. That is, a big amount of high-quality sports service content encourages a high degree of satisfaction and involvement in customer groups, as well as improving the level of final reported sports behavioral intentions as a positive intermediary. The proportion of the effect value of the degree of involvement (effect percent = 52.63%) is slightly higher than that of the satisfaction degree (effect percent = 47.37%) in a further comparative analysis of the influence of the mediation effect, which can judge the impact of the degree of involvement on sports behavioral intention. Satisfaction is not as important as power. As a result, when colleges and universities develop service initiatives to improve students' overall sports behavioral intentions, the value of involvement must be considered. The degree of involvement, particularly in the actual impact path chain, reflects students' cognition and emotional feelings about the importance of sports services in colleges and universities, and to a degree, it can reflect whether the content of sports services provided by the school deviates from the actual sports needs of students (a low level of involvement indicates that students believe the content of sports services provided by the school is not important). This characteristic allows it to partially mediate the beneficial effect of contentment on sports behavioral intention via the H3-H4 pathway, further enhancing the favorable effect of satisfaction on sports behavioral intention.

### 5.4. Influence of Advanced and Basic Sports Services on Sports Behavioral Intention

Multiple studies have found that advanced sports services are more likely than basic sports services to improve behavioral intentions. On the one hand, the correlation analysis reflects this conclusion. Advanced sports services have a stronger correlation between satisfaction, involvement, and sports behavioral intention performance (*r* = 0.680; *r* = 0.421; *r* = 0.407); on the other hand, advanced sports services accounted for a higher proportion of the variance explained in overall sports services (percent variance = 32.113%) in the questionnaire's reliability and validity test. It can be demonstrated that sophisticated sports services have a greater impact on college students' perceptions of sports services. The rationale for this is that basic sports services are concerned with maintaining involvement in sports behaviors, whereas advanced sports services are concerned with improving the quality of those behaviors. Because of the content difference, innovative sports services are able to meet the needs of increasing satisfaction and involvement. A distinct advantage: the purposeful expectation of service content is no longer merely to maintain participation in sports behavior, but to increase the quality of sports behavior, especially for those college students who have acquired regular sports habits. This shift in intentional expectations will have a substantial impact on satisfaction, which reflects psychological expectations and actual needs, as well as participation, which reflects interest and passion, and will, in turn, have an indirect impact on sports activity intentions. It can be seen that, when compared to basic sports services, it is easier to increase investment in advanced sports services to improve the sports behavioral intention of college students who have participated in sports behaviors, in order to increase the frequency, time, and intensity of participation in the future, or to maintain long-term participation and develop the habit of lifelong sports.

RETRACTED

## 6. Study Limitations

In the non-research object control group (college students who have never participated in sports activity), the model's conclusions are quite different, with hypotheses H2 and H3 both being rejected and the level of engagement being unaffected by sports services and sports services. The effect of satisfaction: as a result, the findings of this study can only be applied to college students who have engaged in sports-related activity, and there is no universality. Because the five colleges chosen through purposive selection already have a certain degree of basic sports service provision capability, they can assure that students' involvement in sports behavior is not hindered by physical barriers. If the findings of this study are to be used as a theoretical foundation for increasing investment in modern sports services, the preconditions must be consistent.

## Figures and Tables

**Figure 1:** Hierarchical relationship of sports services in colleges and universities.

**Figure 2:** Hypothetical model.

**Figure 3:** Model path diagram.

**Table 1:** Questionnaire recovery from Hunan Province's five representative universities.

Geographical location	City name	Number of universities	University name	Number of questionnaires
Northern	Changde	6	Hunan University of Arts and Sciences	72
South	Yongzhou	4	Hunan University of Science and Engineering	81
West	Huaihua	4	Huaihua University	67
East	Zhuzhou	10	Hunan University of Technology	113
Central	Xiangtan	14	Hunan University of Science and Technology	149

RETRACTED

**Table 2:** Research variables and measurement dimensions.

Variable	Dimension	Abbreviations	Number of questions
College sport services	Basic sports services	BSS	3
	Advanced sports services	ASS	4
Involvement	Cognitive involvement	CI	3
	Affective involvement	AI	4
Satisfaction	Basic satisfaction	BSAT	3
	Advanced satisfaction	ASAT	4
Sports behavioral intention	Sports behavioral intention	SBI	3

**Table 3:** Reliability and validity test results.

Variable	Item	KMO	Factor loadings	*α*	Total	% Variance
Basic sports services	BSS-1	0.797	0.902	0.784	2.004	28.629
	BSS-2		0.681			
	BSS-3		0.833			
Advanced sports services	ASS-1	0.719	0.731	0.741	2.248	32.113
	ASS-2		0.826			
	ASS-3		0.729			
	ASS-4		0.707			
Cognitive involvement	CI-1	0.769	0.861	0.713	1.868	26.686
	CI-2		0.670			
	CI-3		0.823			
Affective involvement	AI-1	0.803	0.794	0.849	2.645	37.786
	AI-2		0.801			
	AI-3		0.797			
	AI-4		0.859			
Basic satisfaction	BSAT-1	0.844	0.879	0.859	2.131	30.442
	BSAT-2		0.841			
	BSAT-3		0.807			
Advanced satisfaction	ASAT-1	0.771	0.617	0.790	2.554	36.486
	ASAT-2		0.881			
	ASAT-3		0.751			
	ASAT-4		0.913			
Sports behavioral intention	SBI-1	0.904	0.898	0.912	2.592	86.415
	SBI-2		0.946			
	SBI-3		0.944			

**Table 4:** Correlation analysis results.

	BSS	ASS	CI	Ai	BSAT	ASAT	SBI
BSS	1.000	0.413^*∗∗*^	0.361^*∗∗*^	0.302^*∗∗*^	0.624^*∗∗*^	0.316^*∗*^	0.329^*∗∗*^
ASS		1.000	0.371^*∗∗*^	0.421^*∗∗*^	0.357^*∗*^	0.680^*∗∗*^	0.407^*∗∗*^
CI			1.000	0.391^*∗∗*^	0.717^*∗∗*^	0.502^*∗∗*^	0.492^*∗∗*^
AI				1.000	0.539^*∗∗*^	0.830^*∗∗*^	0.381^*∗∗*^
BSAT					1.000	0.467^*∗∗*^	0.614^*∗∗*^
ASAT						1.000	0.696^*∗∗*^
SBI							1.000

Note. ^*∗*^means 0.01 < *P* < 0.05; ^*∗∗*^means *P* < 0.01.

**Table 5:** Model fit index.

*χ*2	df	*χ*2/df	TLI	IFI	CFI	NFI	SRMR	RMSEA
76.681	10	7.668	0.984	0.991	0.993	0.989	0.0375	0.073

**Table 6:** Model path test results.

Assumption	Path	Estimate	S.E.	C.R.	*β*	*R* ^2^	*P*	Conclusion
H1	College sports services ⟶ satisfaction	0.668	0.088	7.617	0.509	0.258	^*∗∗∗*^	Accept
H2	College sports services ⟶ involvement	0.833	0.177	4.702	0.553	0.303	^*∗∗∗*^	Accept
H3	Satisfaction ⟶ involvement	0.407	0.074	5.506	0.514		^*∗∗∗*^	Accept
H4	Satisfaction ⟶ sports behavioral intention	0.439	0.071	6.149	0.362	0.442	^*∗∗∗*^	Accept
H5	Involvement ⟶ sports behavioral intention	0.472	0.086	5.463	0.644		^*∗∗∗*^	Accept

**Table 7:** Bootstrap analysis results of mediating effect.

Influence path	Effect size	Standard error	95% confidence interval		Effect ratio (%)
			Lower limit LLCI	Upper limit ULCI	
Sports service ⟶ satisfaction ⟶ sports behavioral intention	0.235	0.018	0.056	0.154	47.37
Sports service ⟶ involvement ⟶ sports behavioral intention	0.261	0.014	0.036	0.122	52.63
Total effect	0.497	0.033	0.320	0.447	

RETRACTED

## Data Availability

The data used to support the findings of this study are available from the corresponding author upon request.
